# Inhibitory Effect of *Phellinus baumii* Extract on CFA-Induced Inflammation in MH-S Cells through Nuclear Factor-*κ*B and Mitogen-Activated Protein Kinase Signaling Pathways

**DOI:** 10.1155/2021/5535630

**Published:** 2021-10-25

**Authors:** H. M. Arif Ullah, Yuan Yee Lee, Bong-Sik Yun, Sung Dae Kim, Man Hee Rhee

**Affiliations:** ^1^Department of Veterinary Medicine, Cardiovascular Research Institute and College of Veterinary Medicine, Kyungpook National University, Daegu 41566, Republic of Korea; ^2^Department of Neurobiology, University of Utah, Salt Lake, UT, USA; ^3^Division of Biotechnology and Advanced Institute of Environment and Bioscience, College of Environmental and Bioresource Sciences, Jeonbuk National University, Gobong-ro 79, Iksan 54596, Republic of Korea

## Abstract

*Phellinus baumii* is a mushroom utilized as a traditional medicine for a wide range of human ailments, including diabetes, hypertension, hypercholesterolemia, and cancer, in Asia. The purpose of this study was to find out whether *Phellinus baumii* extract (PBE) could reduce inflammation caused by coal fly ash (CFA) in alveolar macrophages (MH-S). The anti-inflammatory effect of PBE was evaluated by measuring the nitric oxide (NO) concentration after the onset of CFA-stimulated inflammation in MH-S cells. Polymerase chain reaction (PCR) was used to examine inflammatory gene expression. Western blotting and immunofluorescence (IF) studies were used to investigate the inflammatory mechanism in MH-S cells. According to our results, the PBE suppressed CFA-induced NO generation in the MH-S cells dose-dependently. Furthermore, PBE inhibited the proinflammatory mediators and cytokines generated by exposure to CFA, including cyclooxygenase 2 (COX-2) and inducible NO synthase (iNOS), interleukin (IL)-1*β*, IL-6, and tumor necrosis factor-alpha (TNF-*α*). Real-time PCR was also used to determine the inhibiting effect of the PBE on proinflammatory factors such as COX-2, iNOS, IL-1*β*, IL-6, and TNF-*α*. Moreover, Western blot was used to assess the effects of the PBE on the nuclear factor-kappa B (NF-*κ*B) and mitogen-activated protein kinase (MAPK) pathways in the CFA-stimulated MH-S cells. The suppressive effect of the PBE on phosphorylated (p)-NF-*κ*B translocation was also investigated using IF analysis. This study showed that the PBE suppressed the CFA-induced inflammation in the MH-S cells by suppressing the NF-*κ*B and MAPK signaling pathways, which suggests its potential usefulness in reducing lung inflammation.

## 1. Introduction

Inflammation is an important aspect of the immune system's defense against damaging stimuli [1, 2]. Dysregulated inflammation is linked to various chronic disorders [3, 4]. Macrophages play an important role in the operation of inflammatory processes, primarily by producing proinflammatory mediators and cytokines such as nitric oxide (NO), inducible NO synthase (iNOS), cyclooxygenase 2 (COX-2), interleukin 1*β* (IL-1*β*), IL-6, and tumor necrosis factor-*α* (TNF-*α*) [4]. Thus, the inhibition of the proinflammatory macrophage activation is considered a vital approach for treating inflammatory disorders.

Particulate matter (PM) in contaminated air is becoming a critical source of health issues [5]. Chronic PM exposure has been linked to chronic inflammatory disorders, particularly severe lung diseases such as chronic respiratory diseases, chronic obstructive pulmonary diseases, asthma, and several types of lung cancer [6–8]. Many pathological and clinical signs of airway inflammatory disorders are linked to excessive production of proinflammatory mediators and cytokines [9, 10]. Alveolar macrophages (MH-S) are immune cells in the immunological regulatory system that are found in the pulmonary alveoli and responsible for upregulating inflammatory mediators caused by exposure to coal fly ash (CFA).

*Phellinus baumii*, a wild fungus, has traditionally been used as healthy food or a folk tonic in East Asia because of its multiple physiological functions, including blood lipid level-lowering, antitumor, antiinfluenza, and antioxidation capacities, and DNA damage-protecting, immune-stimulating, and antidiabetic activities [11–13]. Polysaccharides, polyphenols, and flavonoids, which have a wide spectrum of health benefits and biological activities, have been reported as the principal bioactive ingredients of the *Phellinus* fungus in modern medical research [14–16]. The *Phellinus* fungus includes various yellow polyphenolic chemicals, such as hispidin, that have demonstrated substantial biological effects and have been used to treat diabetes, bacterial, and viral infections, ulcers, and cancer, according to prior studies [11, 17].

Using NO and cell viability assays, as well as the mRNA and protein expressions of proinflammatory cytokines and mediators, we evaluated the anti-inflammatory effects of the *Phellinus baumii* extract (PBE) on CFA-stimulated MH-S cells.

## 2. Materials and Methods

### 2.1. Chemicals and Reagents

RPMI medium for MH-S cells culture, 10% of fetal bovine serum (FBS), 1% of penicillin–streptomycin, Dulbecco's phosphate-buffered saline, 3-(4,5-dimethylthiazol-2-yl)-2,5-diphenyltetrazolium bromide (MTT), coal fly ash (CFA), dimethyl sulfoxide (DMSO) (Sigma-Aldrich, MO, USA); oligo-dT and iNOS, COX-2, IL-1*β*, IL-6, and TNF-*α* primers (Bioneer, Daejeon, Republic of Korea); TRIzol reagent (Invitrogen, CA, USA); proprep (iNtRON Biotechnology, Republic of Korea); bovine serum albumin (BSA) (Thermo Fisher Scientific, Republic of Korea); primary antibodies including phosphorylated (p)-I*κ*B, p-NF-*κ*B, and NOD-like receptor protein 3 (NLRP3), phosphorylated extracellular signal-regulated kinase (p-ERK), total (T)-ERK, phosphorylated c-Jun N-terminal kinase (p-JNK), T-JNK, p-p38, T-p38, *β*-actin, and horseradish peroxidase-linked secondary antibody were used (Cell Signaling Technology, Danvers, MA, USA). A secondary antibody was used for immunofluorescence (IF) (Alexa Fluor 555, IgG Fab2, Molecular Probes). Other reagents were obtained from Sigma-Aldrich.

### 2.2. Preparation of the *Phellinus baumii* Extract (PBE)

We purchased *Phellinus baumii*, which we ground into a coarse powder. We next extracted in 70% ethanol for 24 h using an extractor at 60°C, followed by concentration using the rotary evaporator under reduced pressure. To make a fine powder, the crude extract was frozen overnight at −70°C and lyophilized using a freeze dryer. Finally, the dried extract was ground into a fine powder. During the experiment, the powder was dissolved in DMSO. The concentrate was partitioned using hexane and water, and the hexane-soluble fraction was discarded. The water-soluble fraction was extracted with ethyl acetate. The ethyl acetate-soluble fraction contained yellowish polyphenols of the styrylpyrone class and various oils. Oils were eliminated by washing with chloroform. The remaining polyphenol cluster was dried and powdered for further experiments [18].

### 2.3. Cell Culture and Treatment

The MH-S macrophages were cultured in the RPMI medium and supplemented with 10% heat-inactivated FBS and 1% antibiotics (100 unit/mL penicillin and 100 *μ*g/mL streptomycin), according to our previously described method [19]. The cells were then incubated at 37°C with 5% CO_2_ in a humidified incubator.

### 2.4. Nitric Oxide Assay

The Griess reagents A and B were used to measure NO concentration in accordance with our previous study [7, 19]. In a 24-well plate, MH-S cells were seeded and cultured for 18 h with or without CFA (2.5 *μ*g/mL) and PBE (12.5, 25, 50, and 100 *μ*g/mL) at the doses indicated. 100 *μ*L of Griess reagents were mixed with 100 *μ*L of cell culture supernatants and incubated for 10 min at room temperature. On a microplate reader, the absorbance at 540 nm was measured (VersaMax, Molecular Devices, CA, USA).

### 2.5. Cell Viability Assay

A cell viability experiment was performed as stated using a MTT reagent at 100 *μ*L/well in the culture medium to test the cytotoxicity, as described previously [7, 19]. The supernatants were removed after 2-3 h of incubation at 37°C in 5% CO_2_. The wells were filled with DMSO (100 *μ*L/well) and incubated for 10 min at room temperature with shaking. Finally, the absorbance was measured at 560 nm using a microplate reader (VersaMax, Molecular Devices, CA, USA).

### 2.6. Reverse Transcription Polymerase Chain Reaction and Quantitative Real-Time Polymerase Chain Reaction

Using previously described methods, a polymerase chain reaction (PCR) analysis was done [7, 19]. PBE (12.5, 25, 50, and 100 *μ*g/mL) was applied to cells at the doses indicated for 30 min, followed by 18 h of CFA stimulation (2.5 *μ*g/mL). The RNA was extracted from the cells using the TRIzol reagent.

Two micrograms of total RNA were annealed with oligo-dT at 70°C for 10 min and cooled for 10 min on ice before reverse transcription (RT) in 20 *μ*L of reaction mixture at 42°C for 90 min on a thermocycler. To inactivate the reverse transcriptase, the reaction was stopped at 95°C for 5 min. In a PCR premix, cDNA produced from an RT reaction was used to perform a RT-PCR (Bioneer). On 1% agarose gel stained with ethidium bromide, the PCR products were electrophoresed. ImageQuant LAS 500 was used to visualize the band (GE Healthcare Life Sciences, Republic of Korea). Glyceraldehyde-3-phosphate dehydrogenase (GAPDH) was used as a house keeping gene. SYBR green was used in the real-time PCR. The primer sequences for RT-PCR and real-time PCR are given in Table 1.

### 2.7. Western Blot Analysis

Western blotting was performed with several changes, as described previously [4, 19]. Proteins were isolated from cells, concentrations were determined, and samples were prepared in sodium dodecyl sulfate (SDS) and heated for 5 min. SDS-polyacrylamide gel electrophoresis (SDS-PAGE) was used to separate the samples. The proteins were deposited to the poly (vinylidene fluoride) membranes and blocked for 1 h at room temperature with skim milk (5%). The membranes were washed with washing buffer, tris-buffered saline with Tween (TBST) three times for 10 min each time, and treated overnight at 4°C with the primary antibodies (1 : 1000), namely, p-I*κ*B, p-NF-*κ*B, NLRP3, p-JNK, T-JNK, p-ERK, T-ERK, p-p38, T-p38, and *β*-actin. Furthermore, the membranes were washed with TBST three times for 10 min each time and then incubated with horseradish peroxidase-labeled secondary antibodies (1 : 3000) for 1 h before rinsing with TBST three times for 10 min each. Enhanced chemiluminescence (ECL) solutions A and B (1 : 1 ratio) were used to detect the protein bands in Imager LAS 500 (General Electrics, Boston, MA, USA).

### 2.8. Immunofluorescence Analysis

The immunofluorescence (IF) experiment was performed as described previously [4, 19]. The MH-S cells were rinsed with DPBS and fixed for 10 min in 4% paraformaldehyde. The cells were also permeabilized for 10 min with 0.2% triton X-100 in TBS (TBST) and rinsed three times with TBST for 5 min each time. The samples were blocked for 1 h with 2% BSA before adding rabbit anti-p-NF-*κ*B (primary antibody) overnight at 4°C. MH-S cells were rinsed three times with TBST for 5 min each time. The samples were incubated for 1 h in the dark with a secondary antibody and then washed three times with TBST before being mounted with a Prolong Gold Antifade reagent with 4,6-diamidino-2-phenylindole (DAPI) (Cell Signaling Technology) to observe the nuclei and examined using confocal microscopy (LSM700, Carl Zeiss, Jena, Germany).

### 2.9. Statistical Analysis

The data are represented using the mean and standard error of the mean. One-way analysis of variance was used to establish the statistical significance. The statistical analysis results were considered significant at ^*∗*^*p* values < 0.05, ^∗∗^<0.01, and ^∗∗∗^ <0.001 in comparison to the CFA only group and at ^#^*p* values < 0.001 in comparison to the basal group.

## 3. Results

### 3.1. *Phellinus baumii* Extract Protected against Coal Fly Ash-Induced Nitric Oxide (NO) Generation and Cell Death in the Alveolar Macrophage Cells

NO is a key mediator in the inflammatory process, and its overproduction contributes to the development of inflammatory disorders. The Griess reaction method was used to quantify the NO levels in the murine MH-S in response to CFA stimulation in this investigation. The NO induction was potently reduced by PBE dose-dependently (Figure 1(a)).

Cell vitality was determined using the MTT test, and the results showed that the PBE had no effect on cell toxicity compared with the basal group at the different concentrations used (Figure 1(b)). These findings showed that PBE suppressed the NO generation dose-dependently and that the dosages used were not cytotoxic.

### 3.2. Suppressive Effect of *Phellinus baumii* Extract on Coal Fly Ash-Induced Proinflammatory Cytokines in the Alveolar Macrophage Cells

The levels of the CFA-induced proinflammatory factors were reduced in MH-S after 30 min of pretreatment with PBE. To investigate the anti-inflammatory properties of the PBE, the mRNA expression of iNOS and COX-2, IL-1*β*, IL-6, and TNF-*α* were examined using RT-PCR. Levels of the proinflammatory factors were shown to be reduced dose-dependently (Figures 2(a)–2(f)). This result revealed that the PBE inhibited CFA-induced production of inflammatory cytokines and lowered the mRNA levels significantly.

### 3.3. *Phellinus baumii* Extract Ameliorated the Coal Fly Ash-Induced mRNA Expressions of Proinflammatory Cytokines in the Alveolar Macrophage Cells

To validate the RT-PCR results for proinflammatory factors in the MH-S cells, the mRNA expressions of proinflammatory mediators and cytokines were investigated, and those of proinflammatory factors were tested by real-time PCR. The PBE administration significantly reduced the mRNA expression levels of proinflammatory mediators and cytokines in a dose-dependent manner (Figures 3(a)–3(e)). The real-time PCR results demonstrated that PBE lowered proinflammatory factors in a concentration-dependent manner.

### 3.4. *Phellinus baumii* Extract Inhibits the Activation of the Nuclear Factor-*κ*B (NF-*κ*B) and Mitogen-Activated Protein Kinase (MAPK) Signaling Pathways in the Coal Fly Ash-Treated Alveolar Macrophage Cells

It was hypothesized that the effect of PBE on NF-*κ*B and MAPK signaling played a crucial role in inflammation. CFA activates the inflammatory pathway, and NF-*κ*B and MAPK are critical pathways in the inflammatory cascade. Treatment with PBE considerably decreased the NF-*κ*B phosphorylation and the inhibitor of kappa B (I*κ*B) phosphorylation, whereas CFA markedly enhanced phosphorylation of NF-*κ*B, a transcription factor and inhibitor of kappa B (I*κ*B) in MH-S cells.

NLRP3 was also dose-dependently downregulated after treatment with PBE, especially at 100 *μ*g/mL. In addition, the MAPK pathways, including p-JNK, p-p38, and p-ERK, were also significantly dose-dependently inhibited after treatment with PBE compared with treatment with CFA alone. These results suggest that the pretreatment with PBE significantly inhibited the CFA-induced NF-*κ*B, I*κ*B, NLRP3, ERK, JNK, and p38 activation in MH-S cells (Figures 4(a)–4(g)).

### 3.5. *Phellinus baumii* Extract Inhibited the Translocation of NF-*κ*B in the Coal Fly Ash-Treated Alveolar Macrophage Cells

In CFA-stimulated macrophages, activated p-NF-*κ*B translocation from the cytoplasm to the nucleus was examined using an IF assay to see if PBE's anti-inflammatory effects are mediated through signal transduction cascade of NF-*κ*B. CFA treatment promoted the NF-*κ*B translocation from the cytoplasm to the nucleus, but treatment with the maximum dose of PBE (100 *μ*g/mL) dramatically inhibited p-NF-*κ*B nuclear translocation in activated macrophages (Figure 5). Bay-11 was used as an NF-*κ*B inhibitor. According to the immunostaining result, the anti-inflammatory activities of PBE were linked to its inhibiting properties of the NF-*κ*B phosphorylation signaling cascade.

## 4. Discussion

As medicinal herbs have been widely studied for its anti-inflammatory properties [20, 21], we desire to investigate effective medicinal herbs that have potent medicinal properties. *Phellinus baumii* has long been used as herbal medicine in Asia, particularly China, Korea, and Japan for the treatment of a variety of ailments, including diabetes, hypercholesterolemia, and most notably cancer [11, 22]. Earlier studies showed that PBE can block NF-*κ*B, transcription factor, which is a crucial regulator in the inflammatory cascade. The effects of *Phellinus baumii* on CFA-activated inflammation in the alveolar macrophage cell line were investigated in this work.

The extremely high production of NO related to iNOS synthesis is involved in the inflammatory process [23, 24]. iNOS plays a vital role in releasing NO during the pathophysiology of inflammatory diseases [25, 26]. Moreover, COX-2 is also stimulated by inflammatory stimuli during the inflammatory response [27, 28]. In our study, only the CFA-stimulated group showed upregulation of NO production compared with the basal group, whereas pretreatment with PBE reduced the NO production. The combined treatment with PBE significantly decreased the NO induction (Figure 1(a)).

Endotoxins and cytokines prompted fast alterations in the NO gene expression throughout the inflammation process, which resulted in the de novo synthesis of iNOS and COX-2 pathways [24, 29]. The mRNA expression levels of the proinflammatory mediators such as iNOS and COX-2 and the proinflammatory factors such as IL-1*β*, IL-6, and TNF-*α* were upregulated in the CFA-treated group. By contrast, the combination treatment with PBE significantly downregulated the mRNA levels of the proinflammatory factors (Figures 2(a)–2(f)). These results suggest that PBE has the potential to inhibit proinflammatory factors. Our results also support the previous findings that the iNOS and COX-2 expressions were upregulated in the CFA-stimulated group [19] and that treatment with PBE significantly reduced the protein levels of iNOS and COX-2 (Figures 3(a)–3(e)).

The NF-*κ*B and MAPK signaling pathways were reported to be the key pathways for the inflammatory process [30–32]. The transcription factor NF-*κ*B is a critical regulator in the inflammatory cascade [19]. The MAPK signaling pathway plays an important role in the inflammatory mechanism [33]. Therefore, we examined the anti-inflammatory mechanism of PBE in the macrophage cell line. The protein expression levels of p-I*κ*B, p-NF-*κ*B, NLRP3, p-ERK, T-ERK, p-p38, T-p38, p-JNK, and T-JNK were investigated using Western blotting. For the macrophage MH-S cell line treated with CFA, the activity levels of the NF-*κ*B and MAPK signaling pathways were increased by the CFA treatment, whereas treatment with PBE significantly suppressed the NF-*κ*B and MAPK signaling protein expressions (Figures 4(a)–4(g)). On the basis of our findings, we hypothesized that PBE would decrease I*κ*B and NF-*κ*B phosphorylation, causing the proinflammatory factors to be suppressed.

Furthermore, IF staining revealed that CFA increased the p-NF-*κ*B translocation in the nucleus, whereas PBE (100 *μ*g/mL) and Bay-11 (10 *μ*M) significantly decreased the p-NF-*κ*B translocation from the cytoplasm to the nucleus (Figure 5). A similar result was also found in our previous study [19, 34]. Bay-11 has been reported to have an anti-inflammatory activity that inhibits the phosphorylation of I*κ*B [35]. Our findings suggest that PBE inhibited CFA-stimulated inflammation by reducing the activity levels of NF-*κ*B and MAPK signaling pathways (Figure 6). Only in vitro experiments were performed in this study. Large-scale animal excrement should be performed to reveal the specific mechanism of the action of PBE as an anti-inflammatory agent.

## 5. Conclusion

In conclusion, the anti-inflammatory effects of PBE were established in the CFA-stimulated alveolar macrophages. The findings of this work add to our understanding of CFA-induced inflammatory responses and reveal that PBE may decrease proinflammatory factors expression in MH-S cells. According to our findings, the PBE has potential anti-inflammatory qualities for the regulation of inflammation and could be used as an herbal remedy in the prevention and treatment of numerous inflammatory disorders.

## Figures and Tables

**Figure 1:** Effect of *Phellinus baumii* extract (PBE) on coal fly ash (CFA)-stimulated nitric oxide (NO) generation and cell viability in MH-S macrophages. (a) The cells are divided into six groups, namely, the control (basal), CFA only (2.5 *μ*g/mL), and CFA with PBE (12.5, 25, 50, and 100 *μ*g/mL) groups. The cells are treated with the abovementioned PBE concentrations for 30 min prior to the CFA treatment and incubated for 18 h. The NO level is determined using the Griess reagent method. (b) The MTT reagent method used to perform the cell viability experiment. A 24-well plate is used to seed the cells. All the values from the three independent experiments are expressed as standard error of the mean. ^#^*P* < 0.001 in comparison to the basal group. ^*∗*^*P* < 0.05, ^∗∗^*P* < 0.01, and ^∗∗∗^*P* < 0.001 in comparison to the CFA group.

**Figure 2:** Effect of PBE on CFA-stimulated proinflammatory mediators and cytokines in MH-S macrophages analyzed using reverse transcription polymerase chain reaction (RT-PCR). (a) The mRNA levels of proinflammatory mediators (iNOS and COX-2) and proinflammatory cytokines (IL-1*β*, IL-6, and TNF-*α*) measured after 18 h of CFA (2.5 *μ*g/mL) incubation and GAPDH utilized as a housekeeping gene in RT-PCR. (b–f) The levels of protein expression densitometrically analyzed using ImageJ software. A 6-well plate is used to seed the cells, and the PBE doses of 12.5, 25, 50, and 100 *μ*g/mL are used. All the values from three independent experiments are expressed as standard error of the mean. ^#^*P* < 0.001 in comparison to the basal group. ^*∗*^*P* < 0.05, ^∗∗^*P* < 0.01, and ^∗∗∗^*P* < 0.001 in comparison to the CFA group.

**Figure 3:** Effect of PBE on CFA-stimulated mRNA expression in MH-S macrophages measured using real-time polymerase chain reaction (PCR). (a–e) The mRNA levels of iNOS, COX-2, IL-1*β*, IL-6, and TNF-*α* are measured by quantitative real-time PCR after 18 h of CFA (2.5 *μ*g/mL) incubation. GAPDH is used as a control gene. A 6-well plate is used to seed the cells, and PBE doses of 12.5, 25, 50, and 100 *μ*g/mL are used. All the values from three independent experiments are expressed as standard error of mean. ^#^*P* < 0.001 in comparison to the basal group. ^*∗*^*P* < 0.05, ^∗∗^*P* < 0.01, and ^∗∗∗^*P* < 0.001 in comparison to the CFA group.

**Figure 4:** Effect of PBE on CFA-stimulated nuclear factor-kappa B (NF-*κ*B) and mitogen-activated protein kinase (MAPK) pathways in MH-S macrophages. (a) The protein levels of p-I*κ*B, phosphorylated NF-*κ*B, and NOD-like receptor protein 3, and the MAPK (extracellular signal-regulated kinase, p38, and c-Jun N-terminal kinase) pathway investigated using Western blot after 18 h of CFA (2.5 *μ*g/mL) incubation. As a loading control, *β*-actin was used. (b–g) The expression levels of protein were densitometrically analyzed using ImageJ software. A 6-well plate is used to seed the cells, and the PBE doses of 12.5, 25, 50, and 100 *μ*g/mL are used. All the values from three independent experiments are expressed as standard error of the mean. ^#^*P* < 0.001 in comparison to the basal group. ^*∗*^*P* < 0.05, ^∗∗^*P* < 0.01, and ^∗∗∗^*P* < 0.001 in comparison to the CFA group.

**Figure 5:** Effect of PBE on CFA-stimulated nuclear factor-kappa B (NF-*κ*B) translocation in MH-S macrophages. The cells are seeded on a coated cover slip in a 6-well plate and grouped as follows: basal, CFA (2.5 *μ*g/mL)-induced, CFA with PBE (100 *μ*g/mL), and CFA with Bay-11, inhibitor of phosphorylated (p-NF-*κ*B) groups. The cells are treated with PBE and Bay-11 (10 *μ*M) for 30 min prior to the CFA treatment (2.5 *μ*g/mL) and incubated for 18 h. Immunofluorescence staining is used to examine p-NF-*κ*B nuclear translocation. To visualize the nuclei, the samples are mounted using a Prolong Gold Antifade reagent with DAPI (blue). Confocal microscopy (Zeiss) at ×400 original magnification is used to examine stained cells.

**Figure 6:** Mechanism of action of PBE in CFA-stimulated inflammation in MH-S macrophages.

**Table 1:** Primers were used for reverse transcription polymerase chain reaction (RT-PCR) and real-time PCR analysis.

RT-PCR	Forward primer sequences (5′–3′)	Reverse primer sequences (5′–3′)
iNOS	CCCTTCCGAAGTTTCTGGCAGCAGC	GGCTGTCAGAGCCTCGTGGCTTTGG
COX-2	CACTACATCCTGACCCACTT	ATGCTCCTGCTTGAGTATGT
IL-1*β*	CTGTGGAGAAGCTGTGGCAG	GGGATCCACACTCTCCAGCT
IL-6	GTACTCCAGAAGACCAGAGG	TGCTGGTGACAACCACGGCC
TNF-*α*	TTGACCTCAGCGCTGAGTTG	CCTGTAGCCCACGTCGTAGC
GAPDH	CACTCACGGCAAATTCAACGGCAC	GACTCCACGACATACTCAGCAC
Real-time PCR		
iNOS	GGCAGCCTGTGAGACCTTTG	GCATTGGAAGTGAAGCGTTTC
COX-2	GGCAGCCTGTGAGACCTTTG	GCATTGGAAGTGAAGCGTTTC
IL-1*β*	CAACCAACAAGTGATATTCTCCATG	GATCCACACTCTCCAGCTGCA
IL-6	TCCAGTTGCCTTCTTGGGAC	GTGTAATTAAGCCTCCGACTTG
TNF-*α*	TGCCTATGTCTCAGCCTCTTC	GAGGCCATTTGGGAACTTCT
GAPDH	CACTCACGGCAAATTCAACGGCAC	GACTCCACGACATACTCAGCAC

## Data Availability

The data used to support the findings of this study are included within the article.
